# Advantages of Small Incision Surgery in Thyroid Tumors

**DOI:** 10.1155/2022/7794819

**Published:** 2022-07-11

**Authors:** Wen Feng, Yuan Feng, Qixian Diao, Jian Zhou

**Affiliations:** ^1^Operation Room, Qingdao Hospital of Traditional Chinese Medicine, Qingdao, Shandong 266000, China; ^2^Department of General Surgery II, Qingdao Hospital of Traditional Chinese Medicine, Qingdao, Shandong 266000, China

## Abstract

**Objective:**

Thyroid tumor is a common thyroid disease, and the incidence of complications after traditional thyroid surgery is high, which seriously affects the prognosis of patients. With the development of minimally invasive techniques, small incision surgery has a positive impact on changing the traditional thyroid surgery treatment. However, the gap between small incision surgery and traditional thyroid surgery is unclear, so this meta-analysis was used to evaluate its application value.

**Methods:**

Searching English biomedical databases, including PubMed and Science Network and Chinese major biomedical databases, including CNKI, Wanfang, and Weipu. The keywords of the searched articles are as follows: small incision surgery, traditional thyroid surgery, thyroid tumor treatment, clinical efficacy of thyroid tumor, and surgical treatment, and these keywords are searched individually or in combination to track relevant systematic reviews and literature meta-analysis, and conduct other studies. The retrieval period is from the establishment of the database to January 2022. After extracting the article data, the patients were divided into small incision surgery group and traditional thyroid surgery group due to different intervention methods. The Cochrane risk of bias tool was used to assess the quality of the included literature, and RevMan 5.30 was used for meta-analysis.

**Results:**

A total of 9 articles met the inclusion criteria. There were 369 patients with small incision surgery and 364 patients with traditional thyroid surgery. Compared with traditional thyroid surgery, patients treated with small incision surgery had significant short hospitalization time (MD −2.72, 95% CI (−3.32, −2.12)), less amount of bleeding (MD −15.52, 95% CI (−20.40, −10.65)), short incision length (MD −12.73, 95% CI (−16.29, −9.17)), lower VAS score (MD −2.58, 95% CI (−4.08, −1.08)), and less complications (RR 0.30, 95% CI (0.21, 0.44)).

**Conclusion:**

Compared with traditional thyroid surgery, the results show that small incision surgery can shorten the hospital stay of patients with thyroid tumor, reduce the length of incision, reduce the amount of bleeding and the occurrence of complications, reduce postoperative pain, and have a positive effect on postoperative survival of patients.

## 1. Introduction

Thyroid tumor is a multitumor disease that occurs in the head and neck of humans [1]. The incidence of this disease is often lower in men than in women. The common clinical symptom of thyroid tumor patients is that the mass is located in the front and middle of the neck [2–4]. Due to the influence of tumor mass, it will cause a series of complications in patients, including neck discomfort, dyspnea, hoarseness, and dysphagia, which seriously affects the patient, resulting in a significant decrease in the quality of life of patients [5, 6].

Clinical studies have shown that thyroid tumors include benign tumors and malignant tumors [7, 8]. For a single mass with rapid growth, the possibility of malignancy is high, and the younger the patient's age, the greater the possibility of malignancy. Due to obvious symptoms, patients can generally seek medical treatment in time. Benign thyroid tumors are very common. Thyroid tumors account for about 50% of neck masses. Generally, there are no obvious symptoms. When the tumor is large, it will cause symptoms such as dyspnea due to compression of the trachea, esophagus, and nerves. When the tumor rapidly enlarges with hemorrhage, local swelling and pain will occur, and benign thyroid may become malignant, and the probability of this can generally reach about 10% to 20% [9]. According to the 2018 Global Cancer Statistics Report, thyroid cancer ranks ninth in the world in terms of incidence of cancer, with 567,000 cases (including 194,000 in China), accounting for 3.1% of all cancers. Thyroid cancer has jumped to No. 4 on the list of female malignant tumors in China. Thyroid tumor treatment effect has become the top priority affecting national survival [10, 11].

At present, traditional thyroid surgery is mainly used in the clinical treatment of thyroid tumors in my country. Traditional thyroid surgery can effectively remove the lesions and has a significant clinical effect. However, this surgical method has the disadvantages of large trauma and large intraoperative blood loss [12, 13]. Afterwards, there will be obvious scars, which will affect the patient's physical appearance to a certain extent and increase the patient's psychological burden. With the continuous advancement of medical technology in my country, small incision minimally invasive surgery and traditional thyroid surgery have been used in clinical treatment of thyroid tumor diseases. Minimally invasive surgery has the advantages of good effect, less trauma, less intraoperative blood loss, and postoperative aesthetics, and is recognized by the majority of medical staff and patients [14, 15].

Based on the above reports and cognition of related knowledge, this study aims to evaluate the difference between small incision surgery and traditional thyroid surgery in the treatment of thyroid tumors through meta-analysis, and to provide a theoretical basis for clinical treatment of thyroid tumors.

## 2. Methods

### 2.1. Search Strategy

English biomedical databases, including PubMed and Science Network, and Chinese major biomedical databases, including CNKI, Wanfang, and Weipu were searched. The language is limited to Chinese and English. The keywords of the searched articles are as follows: small incision surgery, traditional thyroid surgery, thyroid tumor treatment, clinical efficacy of thyroid tumor, and surgical treatment, and these keywords are searched individually or in combination to track relevant systematic reviews and literature meta-analysis, and conduct other studies. The retrieval period is from the establishment of the database to January 2022.

### 2.2. Inclusion and Exclusion Criteria

Patients over the age of 25 who meet the diagnostic criteria for thyroid tumors were included. A randomized controlled trial (RCT) comparing minimal incision surgery with conventional thyroid surgery for thyroid tumors was conducted. Outcome indicators include operation time, drainage time, hospital stay, postoperative blood loss, postoperative drainage volume, pain score, and complication rate. Apart from small incision surgery and traditional thyroid surgery, no other interventions were involved in this study. The following will be excluded: studies in animals, children, adolescents, or pregnant women; nonrandomized controlled trials; meeting abstracts; and presence of other interventions beyond the purpose of the study.

### 2.3. Paper Screening and Risk of Bias

Two reviewers independently evaluated the title and abstract of an article to determine whether it was eligible to be selected for the study. If any reviewer believes that the article meets the criteria, the full text will be reviewed. If there is a disagreement about the qualifications of the article, the two reviewers will discuss whether the qualifications of the article can be agreed. If the discussion fails to unify the qualifications of the article, the third reviewer will be used for the decision. If need additional information about the article, the reviewers contact the author of the corresponding article to obtain it. The Cochrane risk of bias tool was used to assess the quality of the included articles and the risk of bias.

### 2.4. Data Extraction

The patients included in this study were divided into a small incision surgery group and a traditional thyroid surgery group. These data were also independently extracted by two reviewers based on pre-established data tables. Demographic data including author name, country, publication time, journal name, and patients were extracted. Outcomes recorded included hospitalization time, amount of bleeding, incision length, VAS score, and complication rate. The two reviewers exchanged data sheets, and differences in extracted data were examined, discussed, and unified.

### 2.5. Statistical Analysis

Percentages and relative risk (RR) or mean difference (MD) with 95% confidence interval (CI) were used to describe the data. The *I*^2^ test is used to test the heterogeneity. If the heterogeneity between studies is small (*P* > 0.1, *I*^2^ < 50%), the fixed-effects model is used to merge the effect sizes; if the heterogeneity between studies is obvious (*P* ≤ 0.1, *I*^2^ ≥ 50%), the random-effects model is used to merge the effect size. Statistical analysis and graphs were performed using the RevMan 5.30 software provided by Cochrane Collaboration. *P* < 0.05 was considered significant difference. Also, the funnel plot is used to analyze/check the risk of publication bias.

## 3. Results

### 3.1. Search Results and Study Characteristics

There were 435 records confirmed from the database, 54 duplicate records were deleted, 381 records were obtained by screening, and 315 records were obtained after excluding 66 low-quality documents, including 129 in English and 186 in Chinese. After reading the full text carefully, articles that did not meet the inclusion criteria, incomplete data and nonrandomized controlled trials were excluded according to the inclusion and exclusion criteria, and finally, 9 available articles were obtained. The specific process is shown in Figure 1.

Nine articles were RCT studies, all of which were comparative studies between small incision surgery and traditional thyroid surgery in China, and three of them were comparative studies between thoracoscopic-assisted neck small incision surgery and traditional thyroid surgery. All articles accurately diagnosed thyroid tumors and met the inclusion and exclusion criteria. There were 369 cases in the small incision surgery group and 364 cases in the traditional thyroid surgery group. The rest of the basic features of this paper are shown in Table 1.

6 articles described random sequence generation, 3 articles did not report random sequence generation, 1 article reported allocation concealment, 7 articles did not report the methods of allocation concealment, 1 article did not perform allocation concealment, only 7 articles reported double-blind, and 2 articles did not report a double-blind method. All articles described outcome assessment bias blinding, complete outcome data bias, and selective reporting bias, 5 articles described other risk bias, and 4 articles did not report other risk bias. The quality assessment results are shown in Figure 2.

### 3.2. Meta-Analysis Results

#### 3.2.1. Hospitalization Time

According to the inclusion and exclusion criteria, a total of 9 articles were included to analyze the effect of small incision surgery and traditional thyroid surgery on the length of hospital stay in patients with thyroid tumors. A total of 369 patients with small incision surgery and 364 patients with traditional thyroid surgery were included. The combined effect size MD was −2.72 (95% CI: −3.32, −2.12; *I*^2^ = 94%) by using the random-effect model, as shown in Figure 3. The comprehensive effect size test result was *Z* = 8.92, *P* < 0.00001. The results of meta-analysis confirmed that there was a statistically significant difference between small incision surgery and traditional thyroid surgery on the length of hospital stay in patients with thyroid tumors.

#### 3.2.2. Amount of Bleeding

A total of 8 articles on intraoperative blood loss in patients with thyroid tumors were included in this article, and the effects of small incision surgery and traditional thyroid surgery on intraoperative blood loss in patients with thyroid tumors were analyzed. Included were 329 patients treated with small incision surgery and 329 patients treated with traditional thyroid surgery. The combined effect size MD was −15.52 (95% CI: −20.40, −10.65; *I*^2^ = 97%), as shown in Figure 4. The comprehensive effect size test result was *Z* = 6.25, *P* < 0.00001. Therefore, the meta-analysis results showed that the effect of small incision surgery and traditional thyroid surgery on intraoperative blood loss in patients with thyroid tumor was statistically significant.

#### 3.2.3. Incision Length

A total of 6 articles were included to investigate the effect of small incision surgery and traditional thyroid surgery on incision length in patients with thyroid tumors. Included were 241 patients treated with small incision surgery and 236 patients treated with traditional thyroid surgery. The analysis results showed that (*P* < 0.00001, *I*^2^ = 100%), indicating that there was no homogeneity in the length of surgical incision between patients treated with small incision surgery and patients treated with traditional thyroid surgery, so a random-effect model was used for joint analysis. The combined effect size MD was −12.73, 95% CI (−16.29, −9.17), as shown in Figure 5. The combined effect size test result was *Z* = 7.02, *P* < 0.00001, so the meta-analysis results suggested that the difference in incision length between small incision surgery and traditional thyroid surgery was statistically significant.

#### 3.2.4. VAS Score

A total of 4 articles were included to investigate postoperative VAS score in patients with thyroid tumors treated with minimal incision surgery versus conventional thyroid surgery. Included were 179 patients treated with small incision surgery and 174 patients treated with traditional thyroid surgery. The analysis results showed (*P* < 0.00001, *I*^2^ = 99%), indicating that there was no homogeneity in postoperative VAS scores between patients treated with small incision surgery and those treated with traditional thyroid surgery, so a random-effect model was used for joint analysis. The combined effect size MD was −2.58, 95% CI (−4.08, −1.08), as shown in Figure 6. The comprehensive effect size test result was *Z* = 3.37, *P*=0.0007, so the meta-analysis results showed that the postoperative VAS score difference between small incision surgery and traditional thyroid surgery was statistically significant.

#### 3.2.5. Comparison of Complications

A total of 9 articles were included to study the postoperative complications of patients with thyroid tumors treated with small incision surgery and traditional thyroid surgery. Included were 369 patients treated with small incision surgery and 364 patients treated with traditional thyroid surgery. The results of the analysis showed (*P*=0.097, *I*^2^ = 0%), indicating that there is a homogeneity of postoperative complications in patients treated with small incision surgery and those treated with traditional thyroid surgery, so a fixed effect model was used for joint analysis. The combined effect size RR was 0.30, 95% CI (0.21, 0.44), as shown in Figure 7. The comprehensive effect size test result was *Z* = 6.14, *P* < 0.00001. Therefore, the meta-analysis results showed that there was a statistically significant difference in postoperative complications between small incision surgery and traditional thyroid surgery.

#### 3.2.6. Publication Bias

The funnel plot is used to check the publication bias of complications. It can be seen that the funnel plot show asymmetry, indicating that there may be publication bias, as shown in Figure 8.

#### 3.2.7. Risk of Bias

Among 9 eligible studies, 6 articles describe that random sequence generation is low risk [18, 19, 21–24], 3 articles were with unclear risk of random sequence bias [16, 17, 20]. 1 article reported allocation hidden bias with low risk [17], 7 articles with unclear allocation hidden bias risk [16, 18–20, 22–24], and 1 article reported that allocation hidden bias was high risk [21]. The blinding of participants and researchers bias of 7 articles was low risk [16–18, 20, 21, 23, 24], and unclear risk in 2 articles [19, 22]. Other bias in 5 article was low risk [18–20, 23, 24] and unclear in 4 articles [16, 17, 21, 22]. Also, all studies have judged to a low risk of bias for incomplete outcome data bias, selective reporting domains bias, and blinding of outcome data, as shown in Figure 9.

## 4. Discussion

Thyroid tumors are the most common tumors in the head and neck, and their incidence is higher in women than in men. The clinical symptoms are a mass in the front and middle of the neck, and some patients also have hoarseness, dysphagia, and dyspnea with swallowing activities. There are many types of thyroid tumors, which are divided into benign and malignant. Generally speaking, a single mass that grows faster is more likely to be malignant, and the younger the thyroid mass, the more likely it is to be malignant. At present, surgery is the main treatment for thyroid tumors. However, patients after traditional neck resection often experience complications such as pain, swelling, discomfort when swallowing, and incision adhesion formation, which seriously affect the quality of life of patients [25, 26]. In recent years, with the continuous development of minimally invasive techniques in clinical practice, endoscopic-assisted neck incision surgery is increasingly used in patients with thyroid tumors. Low-position small incision surgery has a small incision and no needle-eye scars, which is more beautiful than traditional thyroid surgery, so it is favored by more and more female patients [27–30].

The results of this study showed that compared with traditional thyroid surgery, small incision surgery can significantly reduce the length of hospital stay and the length of surgical incision in patients with thyroid tumors, and greatly reduce the amount of intraoperative blood loss, which is similar to the results of existing studies. The possible reasons are as follows: small incision surgery was developed on the basis of minimally invasive cosmetic surgery. It has the advantages of small incision and low blood loss, which greatly reduces the hospitalization time of patients, thereby reducing the burden on the patient's family [31, 32].

Complications after thyroid surgery are the most important factors affecting the survival of patients after surgery. They mainly include pain in the anterior neck area, neck numbness and discomfort, subcutaneous nodules, dysphagia, and incision adhesions. Surgery can significantly reduce postoperative pain, reduce neck numbness and dysphagia, and reduce the incidence of incision adhesions, which is consistent with other similar studies [33, 34]. Therefore, small incision surgery can improve the patient's compliance rate and self-confidence, thereby achieving the recovery of mental health and social function.

This study was limited due to the small sample size analyzed and the insufficient power to analyze the results. In the future, multicenter and large-sample studies should be carried out, and randomized controlled trials should be used to further study the effect of small incision surgery on patients with thyroid tumors.

## 5. Conclusion

In summary, compared with traditional thyroid surgery, small incision surgery can shorten the hospital stay of patients with thyroid tumor, reduce the length of incision, reduce the amount of bleeding and the occurrence of complications, reduce postoperative pain, and have a positive effect on postoperative survival of patients. However, the study has disadvantages such as the small number of patients. In the future, a multicenter, large-sample size approach should be used to further study the effect of small incision surgery on patients with thyroid tumors.

## Figures and Tables

**Figure 1:** Flow diagram of the search, screening, and inclusion process.

**Figure 2:** Literature quality evaluation details.

**Figure 3:** Forest plot of hospitalization time. Comparison of hospitalization time between small incision surgery and traditional thyroid surgery. Statistical method: inverse variance of random-effects model (mean difference (MD) and 95% confidence interval (CI)).

**Figure 4:** Forest plot of amount of bleeding. Comparison of amount of bleeding between small incision surgery and traditional thyroid surgery. Statistical method: inverse variance of the random-effects model (mean difference (MD) and 95% confidence interval (CI)).

**Figure 5:** Forest plot of incision length. Comparison of incision length between small incision surgery and traditional thyroid surgery. Statistical method: inverse variance of the random-effects model (mean difference (MD) and 95% confidence interval (CI)).

**Figure 6:** Forest plot of VAS score. Comparison of VAS score between small incision surgery and traditional thyroid surgery. Statistical method: inverse variance of the random-effects model (mean difference (MD) and 95% confidence interval (CI)).

**Figure 7:** Forest plot of complications. Comparison of complications between small incision surgery and traditional thyroid surgery. Statistical method: the inverse variance of the fixed-effects model (risk ratio (RR) and 95% confidence interval (CI)).

**Figure 8:** Funnel plot analysis of possible publication bias for complications. RR, risk ratio; SE, standard error of the mean.

**Figure 9:** The intensity and distribution of the quality risk of the articles included in the study.

**Table 1:** Basic characteristics of the study articles.

Author	Country	Year	Journal	Experimental group (*n*)	Control group (*n*)
Xi [16]	China	2019	Journal of traditional Chinese and Western medicine	35	35
Guo [17]	China	2020	Guide of China medicine	45	45
Guo [18]	China	2020	Guide of China medicine	51	51
Gao [19]	China	2020	World journal of complex medicine	25	25
Wang [20]	China	2021	Medical information	40	35
Qi et al. [21]	China	2020	Clinical medicine & engineering	40	40
Liu and Jing [22]	China	2021	Clinical medicine	43	43
Wang [23]	China	2021	China continuing medical education	50	50
Zhang [24]	China	2014	Pak J med sci	40	40

## Data Availability

The data used to support the findings of this study are available from the corresponding author upon request.
